# Marriage, Face, and the Body: Human Body Health and the Body Symbols of Hui'an Woman in Southeastern China

**DOI:** 10.1155/2022/2167726

**Published:** 2022-08-05

**Authors:** Meiting Chen, Xiaoxu Zhang

**Affiliations:** ^1^School of Communication, Fujian Normal University, Fuzhou 350117, China; ^2^School of Journalism and Communication, Xiamen University, Xiamen 361000, China; ^3^Huaqiao University, Xiamen 361000, China

## Abstract

The body is not only a physical body but also a communicative body which constructs meaning through communication, and the human body health exerts a considerable influence on self-identity and society. The most fundamental power contained in the communicative body of human constitutes our concept and existing culture. Through in-depth interviews, this paper attempts to analyze the daily microphysical practice of Hui'an women of Xuehua Village in Southeastern China and analyze the meaning of symbol which generates from the body of Hui'an women coming and returning between the husbands' and the natal family. Because of the marriage customs of “extended natal residence marriage,” how the interaction of the human body health continues this special marriage custom and preserves the face of women in this community is shown.

## 1. Introduction

### 1.1. Body as a Medium

From the end of the 20th century to the beginning of the 21st century, a climax of body research emerged in academia, and sociology of body began to become an independent research field. At first, the body was regarded as a physical rather than a social phenomenon. Shilling introduced the body as a “physical object.” Naturalistic views of the body have, since the eighteenth century, exerted a considerable influence on how people have perceived the relationship between the body, self-identity, and society [1]. For example, gender inequality is the direct result of damage of human body health. Turner once summarized the three traditions of body research in “The Body and Society,” namely, taking the body as a set of social practices, conceptualizing the body as a symbol system, and understanding the body as a symbol system representing and expressing the power relations [2]. No matter what kind of body research tradition, it implies the body as a medium, as a carrier of meaning, and as a symbol system. The body cannot be separated from communication, and communication cannot be separated from the body, so the importance of the body in the field of communication research is self-evident. Wittgenstein once said: “The human body is the best picture of the human soul” [3]. It is impossible for any society and culture to separate the body from the symbol system, because members of society need to communicate through the body. Moreover, important political, economic, and cultural issues must be expressed through the body. The body is not only a symbolic system but also a carrier of power. The body increasingly tends to become the core of modern people's sense of self-identity in the highly modern environment [1]. Apparently, the body is indeed a fascinating and profound problem.

The body is not the same as the physical body. O'Neill distinguishes five kinds of bodies: the world body, the social body, the political body, the consumer body, and the medical body [4]. He believes that the communicative body that we have and are thinking about is the total medium of our world, history, culture, and political economy. The opinion originated from Merleau-Ponty, who wrote the following in “Phenomenology of Perception”: “The body is the total medium of the world. Sometimes it is limited to preserve the necessary actions, so it presupposes a biological world around us. And at other times, in the process of clarifying these important actions and developing from their superficial meaning to their metaphorical meaning, the body presents a new core meaning through these actions” [5]. O'Neill also pointed out that we should pay attention to the most basic communicative body as sociologists, which is not only the moral foundation of society but also the moral foundation of any kind of social science practice [4].

While the body has become a hot spot in various philosophical and aesthetic theories, modern communication that starts from the body and eventually ends with the body tends to drive the body out of the territory of human communication. Modern communication technology has not only completely changed the dissemination pattern of human information but also fundamentally changed the function and role of the body in information dissemination [6]. Mass communication tends to ignore the material media in communication, namely, the body. The issue of body is an important field that cannot be avoided after reflecting on the social and historical process of “modernization-modernity.” In fact, human beings mainly used the body as a medium to communicate and exchange with themselves, other human beings, and the surrounding world before the emergence of modern media technology [7]. However, the body as a primitive medium has lost its voice in the field of communication research. Under the ritual view of communication, the media is not limited to the mass media. All information carriers can be called media, and the body as a medium is much earlier than any other medium. McLuhan's classic media view that the media is the extension of the human body explains the extension of the body and its influence. He wrote the following in the preface of “Understanding Media”: “The writing of this book runs through this belief, the purpose is to explore the contours of man reflected by the extension of man's technology” [8]. On his opinion, roads, clothing, houses, currency, clock, and so forth are all extensions of the human body, and the human body is a comprehensive communication medium. To a great extent, our bodies exist for communication, interaction, and creation and evolve themselves due to communication, interaction, and creation [9]. Culture and information are loaded on the body, which is an active carrier. This article attempts to start with the daily microphysical practice of Hui'an woman in Xuehua Village, Huidong District, Fujian Province, and analyzes the symbolic meaning of the Hui'an woman's body, which returns back frequently to the natal family because of the marriage custom of extended natal residence, to reveal how the interaction of the body constructs the social culture of the ocean fishing village.

### 1.2. The Extended Natal Residence Marriage of Hui'an Women

The marriage custom of Hui'an women can be attributed to “extended natal residence marriage” or “delayed transfer marriage.” Strictly speaking, the extended natal residence marriage covers most regions of Hui'an. Generally speaking, the so-called Hui'an women who live in the natal families after getting married mainly refer to the 7 townships in the southeast of Hui'an, which are Chongwu, Shanxia, Tuzhai, Dongling, Jingfeng, Xiaozuo, and Wangchuan. They are connected into one region, and all belong to the coastal area [10]. It is recorded that the married woman lived with her natal family in Xuehua. From then on, the married man sent relative child or his mother to the wife's home to invite her, to come to the husband's home for celebrating holidays or helping in farmwork only during the busy farming season and some important festivals such as Dragon Boat Festival, Mid-Autumn Festival, Winter Festival, and Spring Festival's Eve. The woman can also refuse to return, but she has to on Spring Festival's Eve. This situation continued until their first child was born [11]. Most of the people of Fujian and Guangdong are now of Han nationality, which is a mixed nation. In ancient times, the aborigines of Fujian and Guangdong were ethnic minorities, and their civilization was later than that of the Huaxia nationality in the north. Therefore, more ancient customs were preserved in Fujian and Guangdong. The custom of “extended natal residence marriage” should also be an ancient custom left over from ancient times. Professor Lin believes that although the “extended natal residence marriage” of the Han nationality has the same origin as the “delayed transfer marriage” of the minority nationality, it has been partially changed due to the influence of the feudal society. It is mainly reflected in the oppression of women in the feudal society. Women's status is low. Even if they live in their parents' home for a long time, they must keep their virginity. The husband can beat and scold his wife. The wife cannot rely on her parents' home permanently and cannot return to her husband's home. Therefore, it contributes to their pessimistic suicide. Women in some areas of Huidong live in their parents' home for a long time after marriage, but they need to strictly observe chastity and eliminate any contact with men, which is quite different from women's sexual freedom in ethnic minorities. It can be seen that the “extended natal residence marriage” in some areas of Huidong has its unique form.

This peculiar marriage custom in Huidong area connects Hui'an women with ethnic minorities, which has attracted many scholars to explore the origin of the extended natal residence marriage. Professor Lin of Xiamen University was the first to explore marriage customs in Huidong area. He believes that this custom occurred during the transition period from matrilineal clan society to patrilineal clan society, based on the information obtained during the agrarian revolution and inquiries about his Hui'an friends, as well as relevant newspaper records and historical archives [12]. Engels explains the transition from matriarchy to patriarchy in the book titled “The Origin of Family, Private Property and the State”: “The overthrow of matriarchy is a failure of women with historical significance” [13]. In this way, the extended natal residence marriage, which is the product of institutional changes, can also be seen as the compromised result with a sense of resistance in the process of transition from the matrilineal system to the patrilineal system. Wang holds the same view and believes that no matter what type of extended natal residence marriage, it is mostly related to the matrilineal clan system, and these nationalities also have traces of matrilineal system to varying degrees [14]. Jiang pointed out that the first residents in Huidong area were Minyue people of Baiyue nationality through field investigation and literature review. After mixing with a large number of Han people who immigrated in the Ming Dynasty, they formed the current Huidong residents of Han nationality. This special marriage custom is the product of the combination of the marriage custom of the aboriginal Minyue people and the feudal concept of chastity in the Han culture [15]. Both Han culture and Minyue culture made certain concessions and compromises and experienced a complex process of cultural restructuring: married women lost the social freedom of social contact while living in their parents' home, while men also gave up their husbands' rights for a long time.

However, whether the extended natal residence marriage is part of the Minyue Culture is still unknown. Qiao denies the “relic custom theory” of this marriage custom. From the perspective of function theory, he believes that the marriage custom in each region has its own special causes. The marriage custom in Huidong area is directly related to the local gender division of labor. The extended natal residence marriage enables local women to take into account the interests of their mother's family and husband's family [16]. Wu does not agree with Qiao's negation of the general law of social evolution history. He believes that the extended natal residence marriage not only reflects the system of an extreme patriarchal society but also results from the interaction between the gender division system and the husband's power system [17]. However, in the coastal area near Huidong, the division of labor between men and women is roughly the same; there is no extended natal residence marriage. Guo denies the “relic custom theory” and does not agree with the statement of gender division of labor. Through field investigation and literature review, he points out that Huidong culture has the cultural characteristics of Dan-Min, and the extended natal residence marriage is the product of the intermarriage between Dan-Min and Han people [18]. However, Shi points out that the danists ignored the historical fact that there could not be many Dan-Min in Huidong. In the areas dominated by Huidong people, the extremely rare intermarriage between Dan-Min and Han people could not lead to the extended natal residence marriage [19]. Li, a Taiwanese anthropologist, explains the reasons for the occurrence and existence of the extended natal residence marriage from the perspective of ethnic structure. He believes that, in order to maintain their own traditions, the Huidong people have maintained their own characteristic marriage customs in contrast to the Chongwu people [20].

The later scholars also put forward those opinions such as the theory of combining the extended natal residence marriage from the indigenous Minyue people and the concept of feudal chastity in Han culture, the theory of gender division of labor, and the theory of ethnic interaction. Due to the limited information, those explanations that explain the origin of extended residence marriage in some areas of Huidong cannot be justified completely. After more than 40 years of “transform established habits and social customs,” the extended natal residence marriage still existed firmly in Xuehua. There are two reasons for the continuation: First, it is affected by the long-standing feudal consciousness and old customs. Second, the special gender division of labor in Huidong area is an important factor to preserve the extended natal residence marriage [21]. Because men fish outside all year round, women prefer to help their parents work in their familiar home. Most scholars believe that the economic reasons are very important. Girls are still an important labor force in their parents' family. Marrying out too early will cause economic losses to their parents' family. Therefore, keeping the extended natal residence marriage has become a compromise to meet the interests of both parties. This marriage custom is obviously not necessarily related to ethnic composition. It exists in both ethnic minorities and the Han nationality. Obviously, the marriage custom which exists in both ethnic minorities and Han nationalities has no inevitable connection with ethnicity. It was not until the end of the 20th century that the marriage custom gradually disappeared, because the local economy developed rapidly, especially after the booming of the stone carving industry. What role does the body play in the inheritance and disappearance of the marriage custom of “extended natal residence marriage?”

## 2. Materials and Methods

Xuehua, an assumed name, the field site selected for this study, is a seaside fishing village in southeastern China. It is located between N24°22′∼24°54′ north latitude and E113°53′∼118°59′ east longitude. It belongs to a subtropical maritime monsoon climate zone. Located at the easternmost end of the Chongwu Peninsula, it protrudes over the Taiwan Strait, surrounded by the sea on three sides. Therefore, it is often windy, with an annual average of 6.9 meters per second. The wind is relatively strong from October to February of the following year. The wind speed, wind direction, and windy days in Xuehua are shown in Table 1. As shown in Table 1, November is the month with the highest average wind velocity and the longest continuous windy days in a year, and the maximum velocity, windy days in average, and windy days in sum of November are all in the forefront of the year. The strong wind obviously caused great damage to human body health, especially the skin. As a result, the local Hui'an women (except those under 30) wear a headscarf to guard against the sea breeze all the year round.

The village is divided into four areas for management, the southeast, southwest, northeast, and northwest; Figure 1 shows the panorama of Xuehua [11]. The idea of cherishing every piece of land that can be planted is rooted in the hearts of Hui'an woman in Xuehua because of the scarce arable land. Therefore, even if there is no separate field for planting, the hostess of every household will not miss any available space; see Figure 2. Now the roads extending in all directions integrate Xuehua into the booming economic network of Fuzhou, Xiamen, and other coastal areas, making it more convenient for Xuehua to connect with the outside world.

During the four-month field investigation, the main work for the first two months was to get familiar with the local customs; the old peoples's club in Xuehua was a key turning point. The researcher got to know the hospitable retired clerk, who has many connections in the village and introduced many famous people to the researcher, including the owners of the stone carving factory, the old captains, retired and current cadres, innkeepers, and stone carvers. The researcher slowly built up personal connections through snowballing. In the next two months, the main purpose was to fully develop the in-depth interview part of the research by snowball sampling. A total of 67 people were interviewed from November 2017 to April 2018, including 34 males and 33 females, covering men and women aged from 20 to 90 years and including the main types of local occupations. The interview questions mainly focus on their body health, such as local marriage customs, occupations, and clothing, as well as other daily practices. The male code is M and the female code is F. The basic information of the interviewees is listed in Table 2.

The marked age in this article is the age of interviewee at the time of the interview.

## 3. Field Description and Discussion

Goffman absorbs the principles of theatrical performance and developed his theatrical performance theory, using the metaphor of theatrical performance, such as performer, audience, role, script, “patterns of appropriate conduct,” front stage, and back stage, to describe the ways we present ourselves in daily life, which vividly portrays the details of symbolic interaction between individuals in daily life. The Xuehua Village also seems to be a big stage of the society where everyone in the community shares the accepted values of society. They restraint each others' behaviors in the front stage and try to maintain or control impressions fostered by their performance in a specific situation through adjusting the most obvious physical signals. Hui'an women in particular consciously express themselves and unintentional communication through their bodies, and others in Xuehua are also accustomed to that. Those embodied practice of Hui'an woman in Xuehua who is refusing to return to the husband's home, concealing her face to show her embarrassment, and getting close to her sisters and alienating herself from her husband, imprinted social values, social relationships, and so forth on individuals, forming a unique mystery and charming culture that distinguished Xuehua from other Han communities.

### 3.1. The Female Body That Refused to Return to the Husband's Home

Using the body as a medium, the embodied practice of local women expressed their willingness to refuse to return to the husband's home. Before being married and not having a child, the physical moving between the husband's home and the natal home constructed the legality and special meaning of the extended natal residence marriage and formed a set of predetermined modes of action that refused to return to the husband's home, which Goffman called patterns of appropriate conduct. The Hui'an women in Xuehua were very familiar with this script; they purposely expressed themselves through the patterns of appropriate conduct, playing the female roles prescribed by the Xuehua Villagers, in order to maintain the normal evaluation of them by others. In the summer of 1994, when an American scholar who was doing fieldwork in Xuehua visited a local family, she witnessed the scene of a Hui'an woman avoiding her mother-in-law to call her back to her husband's home.

The oldest daughter in the household, Bbingden, was twenty-six at the time and had been married to her fisherman husband for five years. One evening during my visit, Bbingden's mother-in-law suddenly entered the family courtyard, with her sandals churning up dust as the sound of rubber on tile announced her arrival. She had come to ask Bbingden to spend the night with her son. Bbingden's sister turned to me as the older woman walked past and commented, “she'll refuse to go,” adding that Bbingden would use me as an excuse to explain why she could not traverse the few village paths that led to her husband's home. Sure enough, Bbingden soon appeared out of the lengthening shadows, her headscarf and headpiece tidily in place and her cropped top neatly buttoned down the side. She grabbed my arm and pulled me through the back door and into the street, walking briskly to escape her mother-in-law [22].

Although such a scene has disappeared nowadays, it still exists vividly in the memories of the locals. Returning to or not coming back to the husband's home seems to be a game between wives and husbands. The game marked by the appearance of the female body often ends in the frustration that the husband's family cannot call back the wife. Although the husband's family is often unable to call back the wife, no one tries to omit this seemingly fruitless movement in the process, because not calling the wife back may mean a break between the two parties, which will start a new round of unfamiliar symbolic interaction. Therefore, the patterns of appropriate conduct of refusing to return to the husband's home which includes the husband's family coming to call back the wife and the wife fleeing to avoid returning to the husband's home have been unanimously approved by the performers, the assisting participants, and the audience. It seems that women have the autonomy to refuse to return to the husband's home, but in fact they are just succumbing to the accepted values of society. Woman's avoidance behavior which changes the body of woman from being present to being absent, to avoid direct face-to-face meetings with the husband's family, is a compromise solution to protect the faces of both parties. Face-saving is actually an action of impression finishing and decorating, which is an act that an individual deliberately shows to others in order to make others have a certain impression of himself or herself [23]. Women in Xuehua deliberately used their physical absence to perform well for this conventional drama; they also added another auxiliary role, which was child.

F2: they always asked the children to call the wife, because the husband would not go. Sometimes it's the mother-in-law to call the wife back, and it was best for the children to do that. There was nothing the mother-in-law can do if the bride refused.

F26: My fourth aunt, she was good at escaping. As long as my little aunt called her, she would disappear, as a result my little aunt could not find her. Sometimes it was not until night that she was able to caught her sister-in-law and bring her home. Anyway, bringing sister-in-law home was the task of the two sisters of my father, they must call her back, otherwise they dared not go home.

The patterns of appropriate conduct allow the female body in Xuehua to be properly arranged in daily interactions, maintaining the dignity of both the natal family and the husband's family. Both parties perform themselves in the interaction, play their respective roles, and express etiquette and show goodwill, but behavior that breaks the rules is not allowed. There are historical and practical reasons for the continuation of the extended natal residence marriage in this fishing village near the sea. There is little contact with the outside world because of the closed geographical environment, and it is difficult to be affected by foreign cultures, resulting in a highly closed state of this traditional culture [15]. The lack of labor at home caused by men perennially fishing outside also highlights the female labor force. Significantly, the gender division of labor of “men do the fishing and women do the farming” provides soil for the continuation of the extended natal residence marriage. Both the husband's family and the natal family have acquiesced to this way of living after marriage. Human body health is closely related to division of labor. On the one hand, the extended natal residence marriage has also adapted to the daily production mode and life rhythm of the fishing village from the perspective of functionalism. On the other hand, the husband's home which is unusually unfamiliar for woman due to the extended natal residence marriage belongs to the front stage that requires a complete set of standard expressive equipment as far as micro daily practice is concerned. Hui'an women have three fears (dare to eat, dare not sleep, and dare not speak). Obviously, the natal family belongs to the back stage where woman feel more free is a more comfortable choice, where they do not need to pay attention to their unintentional gesture.

F32: Because I was the oldest in my family, I had to help my natal family. My husband always went out to work. I lived in my natal home until my son was born and I built my own house before returning to my husband's home.

M34: We preferred boys to girls. Men went fishing, and all the work at home was done by women. If you moved to the husband's home as soon as you got married, your natal family would simply lose a very strong labor force. So (her natal home) would not let her go. It would be equivalent to sending a very strong labor force to other family.

F4: I had lived in my natal home for two years. I would return to my husband's home during some important festivals. I returned at night and left in the early morning. It's more comfortable to live in your natal home, you could eat or sleep freely. If you live in your husband's home and you dare not eat enough, then you dare not do anything, which is very inconvenient. Who likes to live there?

However, Chongwu Town, which also relied on fishing for a living and preferred boys to girls, did not have the extended natal residence marriage. This was related to the fact that the women in Chongwu Town had always bound their feet, but the women in Xuehua who had always unbound their feet were skilled in housework and farmwork. Therefore, the interaction of the body between the husband's home and the natal home constitutes a very important nod; the symbolic meaning of the body was constructed during the interaction, which has three key points. First of all, the person who comes to call the Hui'an woman back to the husband's home on a specific holiday shows a gesture of recognizing the marriage, admitting the daughter-in-law, and hoping that the daughter-in-law will return and help. Secondly, the Hui'an woman needs to release a refusal response to the action of calling her back. Finally, the Hui'an woman controls and modifies her behavior by basing on the interpretation of the behavior in her community, and the meaning is contained in the series of social actions. The female body that travels between her husband's and natal homes contains the symbolic meaning of hardworking, strong, and capable woman, and the female body that shows a rejection gesture expresses the symbolic connotation of female shyness recognized by the community.

### 3.2. The Female Body Restricted from Returning to the Husband's Home

Women's physical interactions between the two families connect the daily life of the local residents. However, the extended natal residence marriage is a typical representative of feudalism in official context. Although wives and husbands who have experienced the marriage custom complained strongly, they still followed the traditional custom under strong social pressure. For the locals, this was a custom passed down from ancient times.

For the residents of Xuehua Village, the extended residence of the female body in the natal home releases a well-known normal signal. Once someone tries to break the meaning of this symbol, they will be criticized by the other residents who come to defend the meaning of the symbol. As Goffman said, a person's performance in the personal front can be seen as an effort to show someone's image, and his activities in the region maintain and reflect the accepted values of society [24]. These accepted values of society include two aspects: politeness and decorum. The interactions between two families in Xuehua belong to the front stage, so they should use recognized polite behaviors, which include refusing to return to the husband's home, keeping a distance from their husbands, and going to their natal family as soon as possible, to try their best to show the image of shy, solemn, and modest women in Xuehua to maintain their dignity. In fact, it is a universal impulse to show our own idealized appearance to the world, and performances of individuals always tend to embrace and reflect those values that are officially recognized in society [24]. Therefore, although some individuals are not willing to obey the rules of the extended natal residence marriage in the back stage, they will restrain themselves and others in full accordance with the politeness and decorum required by the extended natal residence marriage in the front stage. The existence of this superficial and disguised agreement comes not only from the historical standard behavior in Xuehua but also from the compliments of the standard behavior that individuals have to express after suppressing their own inner thoughts. The latter reinforces the apparent conformity. When revealing information that contradicts with their idealized image in the front stage, such as they go out to play with their husbands before giving birth, they will have to be faced with the failure of their impression management, which means to confront strong social pressure.

Contrary to the power of refusing to return to the husband's home for the female body, the freedom to return to the husband's home is restricted, and the interaction with the husband is also restricted. Therefore, women do not have the autonomy to control their own bodies, fundamentally speaking. This kind of restraint is reflected not only in the number of contacts but also in all aspects of the female body, among which covering the face and refusing to sleep together with the husband are the most prominent parts. Men and women in Xuehua who are now around 70 years old usually experienced arranged marriages introduced by matchmakers. The procedure introduced by matchmakers is called blind dating. Women's faces are covered with headscarves, while men's faces are unobstructed. Therefore, women are usually able to see their blind date clearly, but men are not. The 73-year-old M12 once met his wife by chance in Chongwu Town after blind dating with her, but he did not recognize her. He told me: “The introduction by the matchmakers was arranged by the parents at the time, there was no affection between the young man and woman at all. Moreover, there was no way to fall in love freely then. I had never contact with my wife before getting married, and no chance to develop romantic love. We didn't see each other for one or two year, so we felt strange. If we have mutual affection, we'll miss and want to meet each other. If the situation is opposite, it doesn't matter if we meet or not”. Obviously, the headscarf that covers the face of a female poses a considerable obstacle to the establishment of an intimate relationship between husband and wife.

F11: Hui'an woman used to wear broad-rimmed bamboo hat and headscarf during marriage, with her head down and her face basically invisible. I often listened to people here telling jokes, husbands and wives here did not know each other. Sometimes there were disputes when selling fish and vegetables in the market. In fact, the two parties in a quarrel turned out to husband and wife, but they didn't know.

M18: The headscarves they wrapped at the time made the faces look relatively smaller. They came late at night with the tightly wrapped headscarves, then started working as soon as they arrived, carrying water until 11:00 pm or 12:00 pm. They were chatting with their sworn sisters before arriving at the husband's home, so it was very late when they came. Some of the husbands slept already, and the wives left early the next day.

M19: After getting married for one, two, or three years, we would not be able to reconcile our relationship here. My wife all sleep standing up without going to bed, she just stood by the bed until dawn, and I told her to go to bed but she insists on not. She didn't allow me to touch her.

Qichang Zeng, a technician of Xiamen University Museum of Humanity, once said: “When the Hui'an Women return to the husband's home on Spring Festival's Eve, they entered the room at dark and left before dawn, because they spent the day with their sworn sisters. Women wore black elaborate headscarves that hung down to their faces. The husband couldn't see the wife's face, therefore a married couple hadn't known each other for a few years. Once a man had been married for eight years, and one day he was drying grains in Tuzhaipo, but when he met his wife, he didn't recognize her, and they knew each other after being told by others” [12]. The black headscarf mentioned by Qichang Zeng was forcibly banned by the government after China's Liberation and was replaced by the yellow hat and blue headscarf wrapping the women's faces, making them look strange and mysterious. We can use front stage to refer to the space of a particular performance. The standard expressive equipment in this space, as a part of the front stage, is called setting [24]. Yellow hat, blue headscarf, and the bowing head (see Figure 3) constitute the settings that women need when they perform in the front stage at the husband's home. This standard expressive equipment shows their posture of shyness, allowing them to complete specific performances in the front stage. However, the face as a primary medium of expression and communication has moral connotations [25], the concealment of faces makes the husband and wife lose important communication channels, and it also strongly expresses the moral posture of women resisting their husbands. While women stand by their husband's bed until dawn to refuse physical touch, they also use the present body to convey the struggle of unwilling to be present (regardless of whether it is true in the heart); the long-term state of inner depression caused damage to their body health. This standard expressive equipment with a sense of resistance is very likely to further deteriorate the relationship between husband and wife, while it deepens the intimate relationship between institutionalized same-sex and nonkin bonds.

### 3.3. The Female Body Constrained by the Institutionalized Same-Sex and Nonkin Bonds

Each culture has its own unique structural context, which allows individuals to deal with interpersonal relationships in different ways. The marine production and lifestyle of the Xuehua Village also promote the formation of special institutionalized same-sex and nonkin bonds. Women's refusal to sleep with their husbands is also closely related to the special local companionship between sworn sisters. Friedman defines this special companionship as same-sex, predominantly nonkin, and same-age cohort relationships formed by groups of women and men. They usually originate in childhood (although that is changing more recently) and tend to incorporate peers from one's own village—neighbors, classmates, workmates, and sometimes children of a parent's dui pnua. The institutionalized same-sex and nonkin bonds are normal in the local society, but they are not homosexual [22]. Male groups are brothers and female groups are sisters in Xuehua. However, the mutual restraint is extremely powerful in female groups.

F2: Sworn sisters went out to do farm work together during the day, and when we came back at night we would talk together and finally all agreed that when the husbands' side called us back on the fifteenth day of the first month, we refused to return. One took the lead and said not to return, others would agree. We promised that no one would go back, and then no one would. If the husbands' side called we back, we would hide ourselves to prevent from being called back, no matter what method was used.

F32: In the past, sworn sisters always arranged the time to leave (to go to our natal home). If the husband was friendly, the wife could come out early and waited for sworn sisters. Some husbands were not friendly (would not let you go), then the sworn sisters waited for you for a long time and got angry.

The importance of face-saving is particularly emphasized in Chinese traditional culture. Benedict attributed Japanese culture to a shame culture, which is different from the Western guilt culture. Its coercive force comes from the external society rather than inner thoughts of everyone. Caring about other people's views of oneself is a prominent feature of the shame culture, and saving one's face to avoid feeling shame is also one of the main reasons why local women obey the extended natal residence marriage. The perception of the individual from sworn brothers and sworn sisters constitutes the main source of the individual's self-concept. Cooley calls this social self-concept, which is determined by the attitude towards the consciousness of the imaginary others, the self-concept in the mirror [26]. We look at our faces, figures, and clothes in the mirror, because our interest lies in these images that belong to us. Similarly, we learn from our imagination what others think about our appearance, demeanor, purpose, actions, character, friends, and so forth, and we are influenced by these thoughts. Facing with the extended natal residence marriage, once women show a gesture of being close to their husbands, they will be ridiculed or isolated by their sworn sisters. The perception that they are ashamed of being close to their husbands is gradually internalized into women's self-identification. But aberrant behavior will occur when the external pressure is weakened. For example, because F2 was serving as a soldier in the local Hui'an militia post, she kept a certain distance from her sworn sisters, weakening the influence from them. Besides, the society at that time was kind of negative for the requirements of the patterns of appropriate conduct of the extended natal residence marriage. F2 told me: “It was a bit relax at that time. Sometimes my husband came by himself, and we would left together, which was a little more avant-garde.” But it could lead to suicide when the external social pressure is too heavy.

The close relationship of sworn sisters is often accused of destroying the intimate relationship between husband and wife. Preliminary Summary of the Implementation of the Marriage Law in Hui'an County from the Fujian Provincial Woman's Federation believes that couple relationships were generally not harmonious, and many couples actually had no relationship because of the arranged marriage and the bad habits of the extended natal residence marriage. Therefore, many women cherish sisterhood and considered it a shame to be closed with their husbands. Friedman's research on sworn sisters in Huidong found that women established an intimate relationship with each other through intimate practices such as eating together, sleeping together, and telling each other secrets. The close relationship between female groups even surpasses the emotional intimacy between husband and wife. On the one hand, it is attributed to the extended natal residence marriage, which gives sworn sisters the space to foster intimacy. On the other hand, the relationships of sworn sisters are more stable to rely on comparison to the unfamiliar husband who has been away all the year round, and this is the same situation in the male groups. In the days when Hui'an woman returned to the husband's home, the sworn sisters walked with each other on the road and promised to go to the natal home as soon as possible; some even promised to keep a distance with their husbands. The back scarves they wore on their heads before liberation were very complicated to take care of. Once they slept with their husbands, they were unable to avoid messy hair, which was easy to be found by sworn sisters when they went to the natal home together. Moreover, the promised time for going to the natal home was only enough for them to do the housework of the husband's family. Therefore the female body is the carrier of relevant information about what they do in the husband's home, revealing information about their psychological and physiological health. They must be cautious of the expression that the body gives off (contextual, nonverbal, presumably unintentional communication).

## 4. Conclusions

The concretization of human subjectivity is the body: the body is both the carrier and the medium of human [27]. In fact, the body is not only the carrier of physiological thing but also the medium of communication. The embodied practice of Hui'an women in Xuehua who are refusing to return to the husband's home, concealing their faces to show their embarrassment, and getting close to their sisters and alienating themselves from their husbands imprinted social values, social relationships, and so forth on individuals, forming the unique mystery and charming ocean culture in Xuehua, which is different from other Han communities. It also reflects the close relationship between human body health and social interaction.

First of all, the patterns of appropriate conduct, such as the husband's family calling and the woman fleeing to avoid returning to the husband's home, make the body of Hui'an woman be properly arranged in the daily interaction to maintain the face of both the natal family and the husband's family, construct the symbolic meaning of friendly interaction between the two parties, express etiquette, and show goodwill. The interaction of the body between the husband's family and the natal family constitutes a very important nod, and the meaning is contained in the patterns of appropriate conduct of refusing to return to the husband's home. The female body showing the rejection gesture expresses the symbolic meaning of shyness, dignity, and modesty of women recognized by the Xuehua Villagers.

Secondly, the extended residence of the female body in the natal family releases a well-known normal signal. Once someone tries to break this symbol of shyness, dignity, and modesty of women, they will be criticized by the other villagers who come to defend the meaning of the symbol, which represents the face and idealized image of the Hui'an woman. In order to maintain better face, women also need to strengthen their position of safeguarding their faces through embodied practices of covering up their faces and refusing to sleep with their husbands.

Finally, the closed sworn sisters often accompany women when they have to return to the husband's home and promise to go to the natal home as soon as possible, and some even agree to keep a distance from their husbands. The female body is the carrier of relevant information about what they do in the husband's home. They must be careful about the information that their body can reveal to avoid being caught by their sworn sisters. At the same time, they strongly prove their close companionship and reiterate their solemness and innocence through collective suicide.

The body is not only a physical body but also a communicative body which constructs meaning through communication, and the human body health exerts a considerable influence on self-identity and society. The most fundamental power contained in the communicative body of humans constitutes our concept and existing culture. In fact, anthropologists pay more attention to physical issues than sociologists, especially the role of the body in conveying culture and meaning in the ritual process. Through the daily performance of the body and the interaction of symbols, Xuehua Villagers have built a special partner relationship, unique marriage customs, and etiquette of “extended natal residence marriage,” as well as the spiritual connotation of women's diligence and courtesy in the marine civilization. As virtual reality, mobile Internet, artificial intelligence, Internet of things, and other new media issues are attracting more and more attention to the communication significance of multiple presence and virtual presence of the body under technical conditions, reexamining the role and significance of human body in the social practice is the logical starting point for returning to the research of the human body in the field of communication. The research on the body in the field of communication needs to be further expanded.

## Figures and Tables

**Figure 1:** Panorama of Xuehua Village (photographed by the authors in 2017).

**Figure 2:** A corner of of Xuehua Village (photographed by the authors in 2017).

**Figure 3:** The Hui'an women in traditional costumes (photographed by the authors in 2017).

**Table 1:** Wind velocity, wind direction, and windy days.

Month	1	2	3	4	5	6	7	8	9	10	11	12
Average vel. (m/s)	8	8	6.9	5.8	5.6	5.4	5.3	4.9	6.6	8.7	9	8.3
Maximum vel. (m/s)	20	20	20	20	28	18	28	32.6	24	24	24	20
Windy days in average	13.6	12.9	10.1	16.2	3.9	1.5	2.4	3.4	6.3	13.2	15.5	14
Windy days in sum	24	21	19	12	12	7	7	9	13	23	22	22
Maximum number of continuous windy days	11	14	15	7	5	3	6	6	6	17	20	19
Dominant wind direction	NNE	NE	NE	NE	NE	SSW	SSW	SSW	NNE	NNE	NNE	NNE

**Table 2:** Basic information of interviewees.

Male code	Age	Occupation	Female code	Age	Occupation
M1	74	Retired cadre	F1	27	Housewife
M2	72	Retired cadre	F2	45	Government staff
M3	38	Self-employed	F3	72	Retired accountant
M4	56	Fishman	F4	46	Self-employed
M5	48	Worker in stone carving factory	F5	22	Teacher
M6	66	Owner of tone carving factory	F6	42	Company employee
M7	73	Retired cadre	F7	40	Company employee
M8	57	Fishman	F8	54	Housewife
M9	68	Ancient architectural painter	F9	42	Teacher
M10	55	Government staff	F10	42	Housewife
M11	50	Teacher	F11	37	Innkeeper
M12	73	Retired loader driver	F12	39	Inn manager
M13	80	Retired cadre	F13	37	Housewife
M14	83	Retired clan chief	F14	60	Housewife
M15	82	Retired cadre	F15	72	Housewife
M16	85	Retired cadre	F16	45	Government staff
M17	93	Retired cadre	F17	38	Housewife
M18	55	Innkeeper	F18	77	Retired cadres
M19	72	Retired veteran	F19	26	Company employee
M20	73	Electrical equipment repairer	F20	50	Housewife
M21	80	Retired cadre	F21	43	Self-employed
M22	76	Retired fishman	F22	68	Housewife
M23	48	Government staff	F23	87	Retired cadre
M24	81	Retired cadre	F24	80	Retired accountant
M25	63	Retired fishman	F25	85	Housewife
M26	62	Retired ship repairer	F26	33	Worker in stone carving factory
M27	62	Retired fishman	F27	45	Worker in stone carving factory
M28	48	Worker in stone carving factory	F28	41	Worker in stone carving factory
M29	29	Manager of stone carving factory	F29	50	Self-employed
M30	49	Worker in stone carving factory	F30	87	Housewife
M31	43	Worker in stone carving factory	F31	84	Housewife
M32	43	Crew	F32	55	Government staff
M33	48	Crew	F33	35	Self-employed
M34	72	Retired teacher			

## Data Availability

The data used to support the findings of this study are available from the corresponding author upon request.
